The article "Brain Magnetic Resonance Imaging Features of Nicotine-Dependent Individuals and Its Correlation with Polymorphisms of Dopamine D Receptor Gene" was published in 2022. Journal: Contrast Media Mol Imaging.

# Brain Magnetic Resonance Imaging Features of Nicotine-Dependent Individuals and Its Correlation with Polymorphisms of Dopamine D Receptor Gene

**DOI:** 10.1155/2022/2296776

**Published:** 2022-08-24

**Authors:** Hongfeng Liu, Lixin Guan, Ying Nie, Qi Li, Jiting Xue, Yong Yang, Shengzhong Rong, Jun Liang, Yanzhong Guan, Fengguo Zhai, Yanhai Ren, Ziyi An, Zesong Dong, Zhixue Han

**Affiliations:** ^1^Mudanjiang Medical University, Mudanjiang 157011, China; ^2^Heilongjiang University of Chinese Medicine, Harbin 150000, China

## Abstract

The aim of this research was developed to provide a scientific basis for individualized prevention, clinical diagnosis, and corrective treatment of nicotine addiction. The objects were 214 cases in the smoke group and 43 cases in the control group. According to the Fagerstrom Nicotine Dependence Test (FTND), the smokers were divided into mild nicotine dependence group (FTND < 6 points, 138 cases) and nicotine severe dependence group (≥6 points, 76 cases). The brain structure in long-term smokers was evaluated by using magnetic resonance imaging (MRI). The nicotine dependence was further analyzed by grouping the included individuals, and some candidate genes related to nicotine addiction were screened by combining with bioinformatics analysis. The family research strategy was adopted to detect nicotine addiction susceptibility genes and their polymorphisms. The MRI imaging results showed that the bilateral thalamus, right parietal, and left lens gram-molecule volume (GMV) were negatively correlated with smoking index and smoking years in the smoking group. The GMV of the posterior cingulate cortex in the severe nicotine dependence group was lower than that of the control group, and the GMVs of bilateral thalamus and bilateral superior limbic gyrus in the mild nicotine dependence group were lower than those of the control group. The gene polymorphism detection showed that rs6275 was highly polymorphic in the target population and the frequency of rs6275-C allele was 53.26%. Therefore, the MRI imaging characteristics suggested that the affected brain regions of smokers and people with varying degrees of nicotine dependence were mainly concentrated in response-related pathways and the limbic system and had cumulative effects on the central nervous system. In addition, the M6275 polymorphism of DRD2 gene was associated with susceptibility to nicotine addiction in Chinese population, and the M6275-C allele had a protective effect on susceptibility to nicotine addiction and smoking initiation.

## 1. Introduction

Smoking is one of the most important risk factors for chronic noncommunicable diseases, causing serious health, economic, and social problems. It is also the world's leading preventable cause of death. Besides hypertension, smoking is the most serious risk factor for the global disease burden [1, 2]. A large number of studies have proved that smoking is the most important risk factor for the occurrence and death of various diseases such as respiratory system, cardiovascular and cerebrovascular system, and nasopharyngeal cancer. Smoking-related diseases account for half of all deaths worldwide each year. China is a country with the highest tobacco consumption rate in the world; the harm of tobacco will be more serious [3]. Currently, more than 1 million people die each year from tobacco-related diseases in China, which is expected to double in 2025 and 2050, respectively, and triple in 2050. Although most smokers have the desire to quit smoking, the majority of smokers who stop smoking usually relapse within a month, and only a very small number of smokers can achieve complete cessation of smoking through personal efforts. It is so difficult to stop smoking and maintain abstinence, mainly because more than 4,000 harmful substances such as nicotine, coal tar, and carbon monoxide in indoor air are released during the combustion of cigarettes. Among them, nicotine drugs are the most important factor of tobacco addiction [4–6]. Long-term intake of nicotine can cause smokers to be forced to take more nicotine to protect and improve dopamine (DA) levels in the brain to protect or obtain pleasure; otherwise, depression and restlessness will occur. In recent years, scientific research has shown that various drugs (such as nicotine, cocaine, and ethanol) that are violated will damage the structure and function of the central nervous system, thereby interfering with its function [7–9]. Therefore, it is necessary to explore the effect of tobacco on brain function and its guidance on smoking cessation [10]. Domestic and foreign studies have found that the regional gray matter structure of smokers is different from that of nonsmokers in the control group, but the differences are not consistent [11]. Most studies found a decrease in regional gray matter volume in smokers, but other studies found an increase in regional gray matter volume and density [12].

The article "Brain Magnetic Resonance Imaging Features of Nicotine-Dependent Individuals and Its Correlation with Polymorphisms of Dopamine D Receptor Gene" was published in 2022. Journal: Contrast Media Mol Imaging.

Since dopaminergic nervous system activity has an extremely important role in nicotine addiction, polymorphisms affecting dopaminergic nervous system function should be prioritized as candidate genes for smoking-related behaviors. All drugs with dependence may exert their pharmacological effects through common neural pathways. This pathway is the mesolimbic dopamine neural pathway, with the ventral tegmental area and nucleus accumbens as its core, and this system is the body's natural reward tether. Nicotine may stimulate the dopaminergic nerves of this nervous system to increase the release of dopamine, thereby exerting the rewarding effect of nicotine, while the withdrawal response is due to the decrease in the stimulation of mesolimbic dopamine neurons [13, 14]. It is found that the content of dopamine D1 receptors in the nucleus accumbens of experimental animals that could be detected by quantitative immunoblotting was significantly higher than that of nonaddicted animals, while the content of dopamine D2 receptors was significantly decreased. Nicotine can induce conformational changes such as sensitization, desensitization, and inactivation of nicotine receptors, and the long-term effects of nicotine can increase the number of receptors. This low sensitivity and high number of nicotine receptors may underlie the development of nicotine tolerance [15, 16]. In order to explore the genetic basis of the occurrence and development of nicotine addiction, we provide scientific basis for individualized prevention, clinical diagnosis, and corrective treatment of nicotine addiction and provide methodological experience for exploring the genetic mechanism of other addictions. In this research, MRI images were used to evaluate the brain structure of long-term smokers who were further grouped according to the degree of nicotine dependence. Combined with bioinformatics analysis methods, some candidate genes related to nicotine addiction were screened. The nicotine addiction susceptibility gene and its polymorphisms were detected by family research strategy, and on this basis, the interaction between gene-gene and gene-environment was further studied, so as to analyze the distribution of environmental risk factors related to nicotine addiction in samples and their impact on genetic studies.

## 2. Materials and Methods

### 2.1. Research Objects

From December 2019 to December 2021, 214 smokers and 43 nonsmokers were enrolled in hospital. The objects enrolled in this research were all of Han nationality and their dominant hand was the right hand. There were 214 cases in the smoke group and 43 cases in the control group. The smoke group was divided into severe group with 76 cases and mild group with 138 cases according to FTND score. In addition, the smoking index (smoking years × number of cigarettes smoked per day/20) and related scales of alcohol consumption were provided. All subjects voluntarily participated in the experiment and had good compliance. The research was approved by ethics committee of hospital, and all subjects signed an informed consent form before the experiment.

The article "Brain Magnetic Resonance Imaging Features of Nicotine-Dependent Individuals and Its Correlation with Polymorphisms of Dopamine D Receptor Gene" was published in 2022. Journal: Contrast Media Mol Imaging.

The inclusion criteria of smokers met the DSM-IV diagnostic criteria for substance dependence that was smoking ≥10 cigarettes per day and smoking years ≥2 years. Exclusion criteria were set as follows: patients with psychotic symptoms or family history of mental disorders; patients with previous history of epilepsy or family history of epilepsy; patients with a history of dependence or behavior (gambling, online game) addiction in addition to alcohol and drugs; those who were taking or have taken benzodiazepines or antipsychotics within 2 weeks; those who had a history of craniocerebral injury, coma, organic brain, or serious physical diseases and a history of intracranial metal implantation or dentures; and those who could not accept MRI examinations. Before the structural image scan, it was confirmed that there were no lesions or structural abnormalities in the brain and they were all right-handed.

### 2.2. Diagnosis Criteria

The Chinese-translated Fagerstrom Test for Nicotine Dependence (FTND) questionnaire was used as the diagnostic standard for nicotine addiction. According to the respondents' answers to the FTND questionnaire, 0∼10 points (FTND score) can be calculated. Fagerstrom et al. divided nicotine dependence into five grades according to the FTND value, as shown in Table 1.

In this research, nicotine addiction was defined as a current smoker with a FTND score of 8–10 (an individual who smoked more than 5 regular cigarettes (or equivalent) per day for at least one year at the time in which we followed an individual). In addition, regular smokers in this research referred to those who smoked more than 5 regular cigarettes per day for at least one year.

### 2.3. Quality Control

The quality control of the whole research process was composed of two parts: the quality control of epidemiological field and the quality control of laboratory analysis. The specific process was shown in Figure 1.

The quality control of genotyping included the quality control of the experimental process and the quality control of genotyping data. For the quality control of the genotype analysis experimental process, the laboratory designated technicians would randomly select 20% of the experimental samples to check the coincidence rate when the genotype identification experiment of a certain polymorphism locus was completed. Only when the genotype coincidence rate reached 100%, will the genotype data of the polymorphism site be considered valid. For quality control of typing data, the experimental gel map would be interpreted and entered by two people. All controversial and inconclusive data would be determined by a second experiment by comparing the two readings and the entered data. Undetermined data were treated as missing.

The article "Brain Magnetic Resonance Imaging Features of Nicotine-Dependent Individuals and Its Correlation with Polymorphisms of Dopamine D Receptor Gene" was published in 2022. Journal: Contrast Media Mol Imaging.

### 2.4. Preprocessing of MRI Images

Magnetic resonance scanner was 3.0 T Magnetom Skyra magnetic resonance scanner; coil: 16-channel head phased array coil. In this research, SPM8 software based on MATLAB platform was used to process 3D T1 structural images for voxel-based morphological analysis (VBM). It mainly included the following steps.

Data format conversion: it should convert the digital imaging and communications in medicine (DICOM) format of original image to the neuroimaging information technology initiative (NIFTI) format. Segmentation structure: the standard brain structure image template under the SPM8 software was adopted to segment the white matter, gray matter, and cerebrospinal fluid of the structure image. Registration and spatial normalization: to reduce the individual differences caused by differences in the brains, the DARTEL software tool was applied to register and normalize the data. First, it should affine the gray matter density map to the gray matter template in standard space.

### 2.5. Statistical Analysis

VBM processing was performed on the three-dimensional T1 structural images to obtain the gray matter volume per voxel of the whole brain. The magnetic resonance experimental data were analyzed using the general linear model of SPM8 software. The general linear model of SPM8 software was used, with age and years of education as covariates, and independent samples *t*-test (*α* = 0.05 as the test level) was used to compare the differences in gray matter volume between the smoke group and the control group. Differences in gray matter volume among the severe group, the mild group, and the normal control group were compared by variance analysis (with *α* = 0.05 as the test level). IBM SPSS Statistics 26 software was used to analyze the difference area of gray matter volume in the control group, the severe group, and the mild group, and their correlations to the average smoking duration, the number of cigarettes per day, the FTND evaluation, and the smoking index (number of smoking years × the count of smoking per day/20) were analyzed using the Spearman correlation analysis. Differences were considered statistically significant when *P* < 0.05 and statistically and extremely significant when *P* < 0.01.

## 3. Results

### 3.1. Basic Clinical Data

The basic information was shown in Figure 2. The average years of education of the smoke group (14.8 ± 2.7) were generally lower than those of the control group (16.2 ± 1.3), and the difference between the two groups was extremely significant (*P* < 0.01). There was still an extremely significant statistical difference in years of education in the smoke group with moderate to severe group (14.1 ± 2.4) and mild group (14.9 ± 2.8) (*P* < 0.01). In terms of gender, men smoked more than women (183/31). In terms of smoking years and daily smoking volume, the severe group lasted longer and smoked more frequently than the mild group, proving that nicotine dependence smoking years were related to smoking volume.

The article "Brain Magnetic Resonance Imaging Features of Nicotine-Dependent Individuals and Its Correlation with Polymorphisms of Dopamine D Receptor Gene" was published in 2022. Journal: Contrast Media Mol Imaging.

### 3.2. Results of Imaging Analysis

Independent samples *t*-test results showed that, compared with the control group, long-term smokers had decreased bilateral thalamus (right thalamus voxels: 1213; left thalamus voxels: 958), bilateral parietal lobes (right supramarginal gyrus voxels: 878, right postcentral gyrus voxels: 671; left supramarginal gyrus voxels: 922), and left lentiform nucleus (putamen voxels: 324) gray matter volume (GMV) (FWE correction, *P* < 0.05, and cluster size >303 voxels). In addition, no regions with elevated GMV were found. Spearman correlation analysis showed that bilateral thalamus, right superior limbic gyrus, and left lenticular nucleus GMV were negatively correlated with smoking index and smoking years, bilateral thalamus was also negatively correlated with daily smoking amount, and bilateral thalamus was negatively correlated with daily smoking amount. The differences were statistically significant (*P* < 0.05). The specific data were shown in Figures 3 and 4.

### 3.3. Different Brain Regions in the Severe Group, the Mild Group, and the Control Group

As shown in Figure 5, ANOVA (Analysis of Variance) showed that there was a statistically significant difference in GMV among the three groups (FWE correction, *F* = 7.999, *P* < 0.05, and cluster size >211 voxels). After the multiple comparisons, the brain regions that differed between groups were identified.

The severe group was compared with the mild group, as shown in Figure 6 (without FWE correction, *P* < 0.05, and cluster size >150 voxels). The GMV of the former left precentral gyrus decreased (*t* = −4.42, *P* < 0.05), and no GMV increased region was found. Spearman correlation analysis found that the left precentral gyrus GMV was negatively correlated with smoking index and smoking years.

The severe group was compared with the control group, as shown in Figure 7. The former was found to be in the posterior cingulate cortex of the limbic lobe (voxels: 391) with decreased GMV (FWE correction, *t* = −4.26, *P* < 0.05, and cluster size >359 voxels), and no areas with elevated GMV were found. Spearman correlation analysis did not find that there was no significant correlation between GMV in posterior cingulate cortex and smoking behavior data (*a* = 0.05, *P* < 0.05).

The article "Brain Magnetic Resonance Imaging Features of Nicotine-Dependent Individuals and Its Correlation with Polymorphisms of Dopamine D Receptor Gene" was published in 2022. Journal: Contrast Media Mol Imaging.

The mild group was compared with the control group, as shown in Figure 8. The GMV of the former bilateral thalamus (right thalamus voxels: 582; left thalamus voxels: 330) and bilateral supramarginal gyrus (right supramarginal gyrus voxels: 373; left supramarginal gyrus voxels: 852) decreased compared with the control group, showing statistically significant differences (*P* < 0.05). No areas of GMV enlargement were found (FWE correction, *P* < 0.05, and cluster voxel size >318 voxels). The Spearman correlation analysis showed that bilateral thalamus and GMV of the right superior limbic gyrus were negatively correlated with smoking index and smoking years and the right thalamus GMV was also negatively correlated with daily smoking.

### 3.4. Differences in Gene Types

Different genotypes had no significant differences in gender, age, height, marital status, educational frustration, and family members' attitudes towards smoking and alcoholism, but there were statistical differences in occupation, cardiovascular history, diastolic blood pressure, and nicotine addiction status (*P* < 0.05). The frequency of rs6275-C allele (*N* = 214) was 53.26%. In random samples without blood relationship, the rs6275 genotype distribution was consistent with Hardy-Weinberg equilibrium (*f* = 1.92, *P*=0.163). One sibling (*N* = 32) was randomly selected from one family, and the genotype distribution of rs6275 was also in line with Hardy-Weinberg equilibrium (*f* = 0.12. *P*=0.873). In pedigree linkage disequilibrium analysis (TDT and TDT-SDT combined analysis), no significant transmission/linkage disequilibrium was detected between nicotine addiction, withdrawal, initiation of smoking, and alcoholism and the rs6275-C allele. The linear regression results of nicotine addiction and early onset smoking were shown in Figure 9.

Both the linear and the logistic regression analyses showed that the rs6275-C allele was significantly and negatively correlated with nicotine addiction susceptibility to early smoking initiation. Compared with individuals with TT genotype, the degree of nicotine T′ dependence was lower in rS6275 C allele carriers, and the partial regression coefficients (B) of CT genotype and CC genotype affecting the degree of nicotine dependence were −0.51 (S.E. = 0.17, *P*=0.0025) and −0.55 (S.E. = 0.20, *P*=0.0052). However, linear regression did not find a significant association between smoking initiation age and the rs6275 C allele. Logistic regression analysis suggested that CT genotype and CC genotype significantly reduced the susceptibility to nicotine addiction (CT genotype: OR = 0.37, *P*=0.043; CC genotype: OR = 0.26, *P*=0.0056). The protective effect of rs6275-C allele on nicotine addiction susceptibility showed a clear dose-effect relationship. The rs6275-C allele also made a relatively lower susceptibility to early initiation of smoking but did not show a significant dose-response relationship (compared with individuals with TT genotype, OR in individuals with CT genotype = 0.63, *P*=0.034; but, among individuals with CC genotype, OR = 0.62, *P*=0.049).

The article "Brain Magnetic Resonance Imaging Features of Nicotine-Dependent Individuals and Its Correlation with Polymorphisms of Dopamine D Receptor Gene" was published in 2022. Journal: Contrast Media Mol Imaging.

## 4. Discussion

There are two common methods for morphological studies of brain structures based on MRI images: region of interest (ROI) studies and voxel-based morphometric measurements (VBM) studies. The ROI method firstly defines a specific area based on the conclusions of previous studies or certain hypotheses and then uses a computer to automatically analyze the defined area. This method is highly subjective and time-consuming and lacks comprehensiveness and repeatability, so the application of the ROI method is limited to a certain extent. The VBM method is proposed by Ashburner and Friston [17]. It is an analysis technology based on the whole brain and is automatically processed by a computer. The local density or volume of gray and white matter is compared in the whole brain changes in white matter density and volume. In this way, the morphological changes of brain tissue can be accurately displayed, so as to understand the damage of brain neurons. VBM performs an overall analysis of the high-resolution anatomical images of the whole brain at the voxel level, without the need to manually set the region of interest, with high objectivity and accuracy. At present, it has been widely used in brain structural changes caused by central nervous system diseases [18].

In recent years, more and more attention has been paid to the effects of smoking on brain structure, especially the relationship between smoking and brain tissue volume or local density. However, previous morphological studies have not reached a consensus and there are few studies on nicotine dependence. Nicotine dependence is a relatively stable feature of tobacco addiction severity [19]. The FTND score can objectively evaluate nicotine dependence and addiction. It also measures people's dependence on smoking from a psychological perspective. This indicator is a reliable one of stable genetic traits associated with smoking. It is also a potential quantitative indicator of anatomical differences between smokers and nonsmokers [20]. Furthermore, grouping all smokers into one group may not reveal fewer distinct brain regions, as people with less exposure to smoking or light dependence on smoking may have an intermediate brain phenotype. Therefore, it divided the smoke group into a severe group (FTND ≥ 6 points) and a mild group (FTND < 6 points) according to the FTND score in this research to determine the nicotine-dependent brain regions and the behavioral differences of smokers, showing a high significance for smoking cessation guidance [21].

The article "Brain Magnetic Resonance Imaging Features of Nicotine-Dependent Individuals and Its Correlation with Polymorphisms of Dopamine D Receptor Gene" was published in 2022. Journal: Contrast Media Mol Imaging.

Research has shown that nicotine is addictive through reward mechanisms, primarily the limbic dopamine system. Nicotine interacts with receptors in the central nervous system, particularly nicotine acetylcholine receptors, with high potency. By activating acetylcholine receptors, nicotine modulates the transmission and release of different central neurotransmitters, thereby causing dependence [22, 23]. Meanwhile, DA is associated with craving and enhancement in nicotine addiction, primarily stimulating DA signaling, amplifying the effects of drugs and drug-related cues, leading to compulsive drug use and addiction [24]. Decreased thalamic volume is associated with nicotine-induced impairment of neurotransmitter modulation, and reduced thalamic gray matter volume promotes related functions. It was found in this research that long-term smokers had reduced gray matter volume in the left lentiform nucleus. Notably, putamen gray matter volume was also negatively correlated with smoking index and smoking years in smokers; that is, the more the smoking in the lifetime, the smaller the putamen volume, which may be a biomarker of the cumulative effect of smoking [25]. Some studies suggest that smokers have a larger core before they start smoking, which may also be one reason why they become heavy smokers. Preexisting differences in GMV predispose individuals to differences in drug use, which may also explain the differences between this research and previous studies [26]. When the nicotine dependence is classified, no differences were found among the three groups in this study, which may indicate that the putamen differences in different nicotine dependence populations are not obvious, but further studies are needed to expand the sample.

A study found that the dopamine receptor type 2 (DRD2) Taq1A polymorphism is associated with tobacco use and smoking behavior, and the association is stronger in men than in women [27]. Since rs6275 is highly polymorphic in this study population, in line with Hardy-Weinberg, in balanced population, the number of available parents of the m6275 heterozygous genotype was also relatively large. It was one of the reasons why TDT and TDT-SDT combined analyses were selected in this research. In addition, TDT analysis utilizes heterozygous genotype parents and their children with diseased status, which does not require evaluation of nondiseased status (i.e., the definition of controls) and avoids confounding due to erroneous evaluation of controls [28]. Although pedigree-based TDT or TDT-SDT analysis can avoid false-positive results due to population confounding, it has low sensitivity for detecting associations. This may be one of the reasons why there is no significant linkage disequilibrium between the rs6275 polymorphism and nicotine addiction susceptibility detected by TDT and TDT-SDT in this sample [29]. Since the samples in this research came from an ideal genetic population, there was no obvious population confounding in the target population. In addition, it adjusted for some individual and environmental factors affecting susceptibility to nicotine addiction in the regression analysis in this research, thus avoiding the confounding effect of environmental factors. In conclusion, results in this research revealed that the rs6275 polymorphism was significantly associated with nicotine addiction susceptibility, suggesting that the DRD2 gene polymorphism had an important effect on the differences in nicotine addiction susceptibility among individuals.

The article "Brain Magnetic Resonance Imaging Features of Nicotine-Dependent Individuals and Its Correlation with Polymorphisms of Dopamine D Receptor Gene" was published in 2022. Journal: Contrast Media Mol Imaging.

## 5. Conclusion

After discussion, this research found that ① smokers and people with different levels of nicotine dependence did have some effects on brain structure. These affected brain regions were mainly concentrated in response-related pathways and the limbic system. ② The MRI imaging suggested that the gray matter volume in some areas of the brain of smokers and nicotine addicts was negatively correlated with smoking index, smoking age, and daily smoking volume, indicating that nicotine had a cumulative effect on the central nervous system. ③ The M6275 polymorphism of DRD2 gene was associated with susceptibility to nicotine addiction in Chinese population, and the M6275-C allele had protective effect on susceptibility to nicotine addiction and smoking initiation. When the nicotine dependence was classified, no differences were found among the three groups in this research, which may indicate that the putamen differences in different nicotine dependence populations were not obvious. In the future, it would be necessary to further expand the samples for research to provide better scientific proof for clinical medicine.

## Figures and Tables

**Figure 1:** Quality control process of the research process.

**Figure 2:** Comparison of basic information of objects between the smoke group (severe group and mild group) and control group. (a) Comparison of basic information between smoke group and control group; (b) comparison of basic situation in smoke group; (c) comparison of smoking status and score in smoke group; (d) comparison of the number of men and women in smoke group and control group. ^#^Compared with severe group, *P* < 0.01.

The article "Brain Magnetic Resonance Imaging Features of Nicotine-Dependent Individuals and Its Correlation with Polymorphisms of Dopamine D Receptor Gene" was published in 2022. Journal: Contrast Media Mol Imaging.

**Figure 3:** Impact result display. Blue areas are changes in the GMV brain area.

**Figure 4:** Imaging analysis results of different brain regions between smoke group and control group. (a) Comparison of gray matter volume between smoke group and control group (the bilateral thalamus was marked, the left putamen was marked as (b), the right parietal was marked as (c), and the left supramarginal gyrus was marked as d); (b) correlation between GMV in different brain regions of smoke group and control group and smoking behavior. ^*∗*^Compared with control group, *P* < 0.05.

**Figure 5:** ANOVA analysis of severe group, mild group, and control group. ^*∗*^Compared with control group, *P* < 0.05; ^#^compared with severe group, *P* < 0.05.

**Figure 6:** Comparative analysis of severe group and mild group. (a) Comparison of GMV in the left precentral gyrus; (b) correlation analysis between the GMV of different brain regions and smoking behavior between the two groups (dotted line is the correlation trend line). ^#^Compared with severe group, *P* < 0.05.

**Figure 7:** Comparative analysis of the severe group and the control group. (a) Comparison of GMV in the posterior cingulate cortex; (b) correlation analysis between the GMV in different brain regions of two groups and smoking behavior (the dashed line is the correlation trend line). ^*∗*^Compared with control group, *P* < 0.05.

**Figure 8:** Comparison of mild group and control group. (a) Comparison of gray matter volume between mild group and control group (a∼d referred to the bilateral thalamus, the left putamen, the right parietal, and the left supramarginal gyrus, respectively); (b) correlation analysis of differential brain area GMV with smoking status. ^*∗*^Compared with control group, *P* < 0.05.

**Figure 9:** Regression analysis between nicotine addiction and early onset smoking and rs6275 genotype. (a) Linear regression between nicotine addiction and early initiation of smoking group. (b) logistic regression analysis of nicotine addiction and early initiation of smoking group. ^*∗*^Compared with severe group, *P* < 0.05; ^#^compared with severe group, *P* < 0.01.

**Table 1:** Fagerstrom degree of nicotine dependence.

Score	Nicotine dependence level
0∼2	Very low
3∼4	Low
5∼6	Medium
7∼8	High
>8	Very high

## Data Availability

The data used to support the findings of this study are available from the corresponding author upon request.

## References

[1] Cross S. J., Linker K. E., Leslie F. M. (2017 Jan 2). Sex-dependent effects of nicotine on the developing brain. *Journal of Neuroscience Research*.

[2] Lin F., Wu G., Zhu L., Lei H. (2015 Jul). Altered brain functional networks in heavy smokers. *Addiction Biology*.

The article "Brain Magnetic Resonance Imaging Features of Nicotine-Dependent Individuals and Its Correlation with Polymorphisms of Dopamine D Receptor Gene" was published in 2022. Journal: Contrast Media Mol Imaging.

[3] Peng P., Li M., Liu H. (2018 May 24). Brain structure alterations in respect to tobacco consumption and nicotine dependence: a comparative voxel-based morphometry study. *Frontiers in Neuroanatomy*.

[4] Shi Y. Y., Zhang Y., Cheng J. L., Zhu C. D., Xu K., Wang W. J. (2019 Mar 5). [Study on the mechanism of brain damage based on structural covariant network to evaluate the brain structure of nicotine addicts]. *Zhonghua Yixue Zazhi*.

[5] Weng J. C., Huang S. Y., Lee M. S., Ho M. C. (2021 May). Association between functional brain alterations and neuropsychological scales in male chronic smokers using resting-state fMRI. *Psychopharmacology (Berl)*.

[6] Wetherill R. R., Jagannathan K., Hager N., Childress A. R., Rao H., Franklin T. R. (2015 Jun 4). Cannabis, cigarettes, and their Co-occurring use: disentangling differences in gray matter volume. *The International Journal of Neuropsychopharmacology*.

[7] Perez Diaz M., Pochon J. B., Ghahremani D. G. (2021 Aug 20). Sex differences in the association of cigarette craving with insula structure. *The International Journal of Neuropsychopharmacology*.

[8] Roh S. (2018 Jan). Scientific evidence for the addictiveness of tobacco and smoking cessation in tobacco litigation. *J Prev Med Public Health*.

[9] Shen Z., Huang P., Wang C. (2019 Aug). Interactions between monoamine oxidase A rs1137070 and smoking on brain structure and function in male smokers. *European Journal of Neuroscience*.

[10] Sun Y., Liu L., Feng J. (2017 Mar 27). MAOA rs1137070 and heroin addiction interactively alter gray matter volume of the salience network. *Scientific Reports*.

[11] Jankovic M. P., Kaufmann M., Kindler C. H. (2008 May). Active research fields in anesthesia: a document co-citation analysis of the anesthetic literature. *Anesthesia & Analgesia*.

[12] González-Alcaide G., Calafat A., Becoña E., Thijs B., Glänzel W. (2016 Sep). Co-citation analysis of articles published in substance abuse journals: intellectual structure and research fields (2001-2012). *Journal of Studies on Alcohol and Drugs*.

[13] Yadav P., Ellinghaus D., Rémy G. (2017 Aug). Genetic factors interact with tobacco smoke to modify risk for inflammatory bowel disease in humans and mice. *Gastroenterology*.

[14] Feki S., Bouzid D., Abida O. (2017 Nov). Genetic association and phenotypic correlation of TLR4 but not NOD2 variants with Tunisian inflammatory bowel disease. *Journal of Digestive Diseases*.

[15] Sadaghiani S., Ng B., Altmann A. (2017 Oct 4). Overdominant effect of a CHRNA4 polymorphism on cingulo-opercular network activity and cognitive control. *Journal of Neuroscience*.

The article "Brain Magnetic Resonance Imaging Features of Nicotine-Dependent Individuals and Its Correlation with Polymorphisms of Dopamine D Receptor Gene" was published in 2022. Journal: Contrast Media Mol Imaging.

[16] Marees A. T., Hammerschlag A. R., Bastarache L. (2018 Jul 1). Exploring the role of low-frequency and rare exonic variants in alcohol and tobacco use. *Drug and Alcohol Dependence*.

[17] Ashburner J., Friston K. J. (2000 May). Voxel-based morphometry—the methods. *NeuroImage*.

[18] Shen Z., Huang P., Wang C., Qian W., Yang Y., Zhang M (2018). Cerebellar gray matter reductions associate with decreased functional connectivity in nicotine-dependent individuals. *Nicotine & Tobacco Research*.

[19] Mackey S., Allgaier N., Chaarani B. (2019 Feb 1). Mega-analysis of gray matter volume in substance dependence: general and substance-specific regional effects. *American Journal of Psychiatry*.

[20] Laudenbach M., Tucker A. M., Runyon S. P., Carroll F. I., Pravetoni M. (2015 Nov 17). The frequency of early-activated hapten-specific B cell subsets predicts the efficacy of vaccines for nicotine dependence. *Vaccine*.

[21] Chaarani B., Kan K. J., Mackey S. (2019 Jul). Low smoking exposure, the adolescent brain, and the modulating role of CHRNA5 polymorphisms. *Biological Psychiatry: Cognitive Neuroscience and Neuroimaging*.

[22] Chye Y., Mackey S., Gutman B. A. (2020 Nov). Subcortical surface morphometry in substance dependence: an ENIGMA addiction working group study. *Addiction Biology*.

[23] Matos-Ocasio F., Espinoza V. E., Correa-Alfonzo P., Khan A. M., O’Dell L. E. (2021 Apr 1). Female rats display greater nicotine withdrawal-induced cellular activation of a central portion of the interpeduncular nucleus versus males: a study of Fos immunoreactivity within provisionally assigned interpeduncular subnuclei. *Drug and Alcohol Dependence*.

[24] Bullock K., Cservenka A., Ray L. A. (2017 May). Severity of alcohol dependence is negatively related to hypothalamic and prefrontal cortical gray matter density in heavy drinking smokers. *The American Journal of Drug and Alcohol Abuse*.

[25] Arvin M. C., Jin X. T., Yan Y. (2019 May 29). Chronic nicotine exposure alters the neurophysiology of habenulo-interpeduncular circuitry. *Journal of Neuroscience*.

[26] Cao Z., Ottino-Gonzalez J., Cupertino R. B. (2021 Sep). Mapping cortical and subcortical asymmetries in substance dependence: findings from the ENIGMA Addiction Working Group. *Addiction Biology*.

[27] Munafò M. R., Timpson N. J., David S. P., Ebrahim S., Lawlor D. A. (2009). Association of the *DRD2* gene Taq1A polymorphism and smoking behavior: a meta-analysis and new data. *Nicotine & Tobacco Research*.

[28] Philibert R. A., Beach S. R. H., Gunter T. D., Brody G. H., Madan A., Gerrard M. (2010 Mar 5). The effect of smoking on MAOA promoter methylation in DNA prepared from lymphoblasts and whole blood. *Am J Med Genet B Neuropsychiatr Genet*.

The article "Brain Magnetic Resonance Imaging Features of Nicotine-Dependent Individuals and Its Correlation with Polymorphisms of Dopamine D Receptor Gene" was published in 2022. Journal: Contrast Media Mol Imaging.

[29] Lutz S., Yip W. K., Hokanson J., Laird N., Lange C. (2013 Feb 28). A general semi-parametric approach to the analysis of genetic association studies in population-based designs. *BMC Genetics*.

